This article has been retracted.

# TGF-β1 Regulation of Estrogen Production in Mature Rat Leydig Cells

**DOI:** 10.1371/journal.pone.0060197

**Published:** 2013-03-29

**Authors:** Man-Li Liu, Huan Wang, Zong-Ren Wang, Yu-Fen Zhang, Yan-Qiu Chen, Fang-Hong Zhu, Yuan-Qiang Zhang, Jing Ma, Zhen Li

**Affiliations:** 1 Department of Traditional Chinese Medicine, Xijing Hospital, the Fourth Military Medical University, Xi'an, People's Republic of China; 2 Department of Human Anatomy and Histology and Embryology, the Fourth Military Medical University, Xi'an, People's Republic of China; 3 Department of Dermatology, Tangdu Hospital, the Fourth Military Medical University, Xi'an, People's Republic of China; The University of Tennessee Health Science Center, United States of America

## Abstract

**Background:**

Besides androgens, estrogens produced in Leydig cells are also crucial for mammalian germ cell differentiation. Transforming growth factor-β1 (TGF-β1) is now known to have multiple effects on regulation of Leydig cell function. The objective of the present study is to determine whether TGF-β1 regulates estradiol (E_2_) synthesis in adult rat Leydig cells and then to assess the impact of TGF-β1 on Cx43-based gap junctional intercellular communication (GJIC) between Leydig cells.

**Methodology/Principal Findings:**

Primary cultured Leydig cells were incubated in the presence of recombinant TGF-β1 and the production of E_2_ as well as testosterone (T) were measured by RIA. The activity of P450arom was addressed by the tritiated water release assay and the expression of *Cyp19* gene was evaluated by Western blotting and real time RT-PCR. The expression of Cx43 and GJIC were investigated with immunofluorescence and fluorescence recovery after photo-bleaching (FRAP), respectively. Results from this study show that TGF-β1 down-regulates the level of E_2_ secretion and the activity of P450arom in a dose-dependent manner in adult Leydig cells. In addition, the expression of Cx43 and GJIC was closely related to the regulation of E_2_ and TGF-β1, and E_2_ treatment in turn restored the inhibition of TGF-β1 on GJIC.

**Conclusions:**

Our results indicate, for the first time in adult rat Leydig cells, that TGF-β1 suppresses P450arom activity, as well as the expression of the *Cyp19* gene, and that depression of E_2_ secretion leads to down-regulation of Cx43-based GJIC between Leydig cells.

## Introduction

Leydig cells situated in the testicular interstitium are the main sites of testosterone production [1]. It has become increasingly clear that in the adult testis besides androgens, other steroid hormones commonly synthesized by Leydig cells and the germ cells, estrogens [2], also play an important role in the development, growth and differentiation of the male reproductive system and maintenance of spermatogenesis [3]. In particular, the demonstration that spermatogenesis is impaired in mice lacking aromatase or the estrogen receptor α (ERα) has shed new light on the role for estrogen in male reproduction [4]. Concomitantly, the discovery of mutations in both the human ERα and aromatase genes [5], [6] has reinforced the idea that estrogen plays a key role in the human male reproductive system.

Leydig cell estradiol (E_2_) is converted from testosterone (T), catalyzed by the microsomal enzymatic complex termed cytochrome P450 aromatase (P450arom), encoded by the single-copy *Cyp19* gene. Despite the presence of aromatase in germ cells in several species, including the mouse, rat, brown bear, bank vole, rooster and man [7], it is worth noting that Leydig cells in the adult testis have also been identified as the major sites of expression of this enzyme [8], which has been shown to be controlled by various factors, such as LH, cyclic cAMP and testosterone, together with other paracrine factors produced by germ cells, such as TNF-α and TGF-β1 [9]. Aromatase transcription occurs via the alternative use of nine distinct tissue-specific promoters located in the first exon of the *Cyp19* gene [10], and promoter PII is the principal promoter active in rat Leydig cells [11]. This promoter contains several cAMP response element (CRE)-like motifs that mediate the effects of the cAMP transduction pathway that potentiates aromatase gene expression and activity. In Leydig cells, both nuclear receptor steroidogenic factor-1 (SF-1) [12] and liver receptor homologue-1 (LRH-1) are able to activate aromatase transcription by binding to the aromatase promoter PII [13]–[14]. Therefore, transcriptional regulation of *Cyp19* is a major mechanism controlling the activity of aromatase which affects E_2_ synthesis. Several lines of evidence suggest a crucial role for TGF-β1 in regulation of Leydig cell function. For instance, TGF-β1 has been shown to inhibit testosterone secretion [15], to suppress proliferation of Leydig cells [16] and to be involved in the morphological differentiation of immature Leydig cells into the adult form [17]. TGF-β1 has also been found to regulate aromatase expression in a tissue-specific manner. It increases aromatase mRNA levels and activity in osteoblast-like cells, THP-1 cells and the leukaemic cell line FLG29.1 [18]–[19]. However, in germ cells [20], granulosa cells [21] and trophoblast cells [22], TGF-β1 suppresses aromatase gene expression. So far, its role in regulating the expression of *Cyp19* and aromatase activity in Leydig cells is not clear.

Gap junctional intercellular communication (GJIC) directs the exchange of small molecules, including ions, second messengers, and other metabolic precursors less than 1 kDa, between adjacent cells, and this function is mainly mediated by proteins called connexins (Cx) [23]. GJIC between testicular cells is also essential for the initiation and maintenance of spermatogenesis [24]; it is also involved in several cellular processes including control of cell proliferation and differentiation [25]. To date, Cx43 is the only Cx detected in Leydig cells of different species [24], and it forms the gap junctions between them. The regulation of Cx43 expression by estrogen has been reported in human myometrium, rat cardiomyocytes and rat prostate [26]–[28]. The rat Cx43 promoter contains several sequences resembling half the palindromic estrogen response elements (half-EREs), which are functional when co-transfected with estrogen receptor cDNA into HeLa cells [29]. In addition, it has been demonstrated that estrogens in osteocyte and mouse embryonic stem cells, also bound to membrane ERα, induce activation of phosphatidylinositol 3-kinase (PI3K)/Akt, and that one of the tyrosine kinases, PI3K/Akt, participates in the up-regulation of Cx43 [30]–[31]. However, the effect of E_2_ on GJIC in Leydig cells and their only gap-junctional connexin Cx43 has not been studied.

To determine whether TGF-β1 regulates E_2_ synthesis in adult rat Leydig cells and to assess the role of E_2_ and TGF-β1 in GJIC between Leydig cells, in the present study we have examined the effects of TGF-β1 on Leydig cell E_2_ synthesis and aromatase activity. The probable function of E_2_ and TGF-β1 in Cx43-based GJIC between rat Leydig cells was also investigated.

## Materials and Methods

### Ethics Statement

The Ethics Committee for Animal Experiments of the Fourth Military Medical University approved all animal work (Permit number: 08014) and the experimental protocols strictly complied with the institutional guidelines and the criteria outlined in the “Guide for Care and Use of Laboratory Animals”. All surgery was performed under sodium pentobarbital anesthesia.

### Isolation and culture of rat Leydig cells

Male SD rats were sacrificed at 3 months of age and the testes were decapsulated under aseptic conditions. Leydig cells were isolated by enzymatic digestion and purified on a continuous Percoll gradient as described previously [32]. Briefly, the testes were incubated for 20 min in culture medium containing 0.25 mg/ml collagenase (Type II, Sigma) in a shaking water bath at 34°C. Separated cells were filtered through two layers of nylon mesh (100 µm pore), centrifuged at 250 g and re-suspended in 55% isotonic Percoll. Following density gradient centrifugation at 20,000 g for 60 min at 4°C, Leydig cell fractions with densities between 1.070–1.088 g/ml were collected from the Percoll gradient. The cells were washed twice with Hanks' buffered saline solution and then cultured in a 37°C, 5% CO_2_ humid incubator in DMEM-F12 for further studies. The purity of Leydig cells was assessed by histochemical staining of 3β-HSD and viability was determined by trypan blue exclusion. The purity was 90–95% and viability was 95–98%.

### Radioimmunoassay of E_2_ and T

Culture medium with TGF-β1 (final concentrations of 1, 2, 5, 10 ng/ml according to previous studies [17], [33]–[35]) was collected and the production of E_2_ and T was measured by employing a commercially available radioimmunoassay kit (Beijing North Institute of Biological Technology, China), in accordance with the manufacturer's instructions. All measurements were repeated three times independently, and data were presented as mean ± standard deviation (SD).

### Aromatase activity determination

The catalytic activity of aromatase in Leydig cells was assayed by the formation of tritiated water from [1β-^3^H]-androstenedione as described previously [36]. Briefly, TGF-β1-treated Leydig cells were incubated with 20 nM 1β-^3^H-androstenedione (New England Nuclear Research Products, Boston, MA, USA) in serum-free medium for 6 h. Incubations were conducted in an identical fashion in the absence of cells to establish background values. Then the medium (600 µl) was extracted with 1,500 µl of ice-cold chloroform and centrifuged at 12,000 g at 4°C for 1 min. The aqueous phase was transferred to a vial containing 400 µl dextran-coated charcoal to remove the residual labelled and unlabelled steroids. The mixture was vortexed for 10 s and centrifuged at 15,000 g at 4°C for 15 min. The supernatant was decanted, mixed with scintillation fluid and counted in a beta-spectrometer; thus, tritiated water formed during the aromatization of [1-^3^H]-androstenedione to estrogen was determined by measuring the radioactivity in the supernatant. Aromatase activity was expressed as rate of incorporation of tritium into water per mg protein per h for Leydig cells. Each experiment was conducted in triplicate and was repeated at least two times to ensure that the results were quantitatively reproducible.

### Western blotting

Western blotting was performed by following a routine protocol. Briefly, Leydig cells were washed with PBS and scraped into 200 µl sodium dodecyl sulfate (SDS) electrophoresis sample buffer (10 mM Tris, pH 6.8, 15% w/v glycerol, 3% w/v SDS, 0.01% w/v bromophenol blue and 5% v/v 2-mercaptoethanol). Then cell lysates were sonicated (60 Hz, 10 s for 3 times) and heated for 10 min at 95°C. Protein samples were separated by 10% SDS-polyacrylamide gel electrophoresis (SDS-PAGE) and transferred to a nitrocellulose membrane. The blotting membranes were blocked with 5% w/v non-fat milk and probed with rabbit anti-Cyp19 (1∶400 dilution, Sigma-Aldrich), mouse anti-Cx43 (1∶200 dilution, Santa Cruz Biotechnology) or rabbit anti-β-actin (1∶400 dilutions, Sigma-Aldrich). After being washed, the membranes were incubated with horseradish peroxidase-conjugated anti-mouse IgG (1∶3,000 dilution, Sigma-Aldrich) for 1 h at room temperature. The bound antibodies were visualized by an electric control loading system (Amersham Biosciences). Semi-quantitative densitometric analysis of Western blotting was performed by Image J software (NIH, Bethesda, USA).

### Real-time RT-PCR

Total RNA was extracted from rat Leydig cells (2×10^6^) using the RNeasy mini kit (Qiagen, Hiddens, Germany) according to the manufacturer's instructions. Routine Dnase (Ambion, Austin, TX, USA) treatment was performed before reverse transcription. First strand cDNA was synthesized from 1 µg RNA with the Omni RT kit (Qiagen). Real-time PCR was set up with the Corbett Rotor-gene TM 6000 (Corbett, Sydney, Australia) by using SYBR Green (Sigma-Aldrich). Primer sequences were as follows: *Cyp19*, 5′-ggtaaattcattgggcttgg-3′ and 5′- cctgtcgtggtcttggtca-3′; G*apdh*, 5′-cgaccacctttgtcaagctca-3′ and 5′-aggggtctacatggcaactg -3′. The *Gapdh* from the same exacts were used as internal control. The amount of *Cyp19* was normalized to the G*apdh* value. Data were calculated from the mean of three experiments.

### Immunofluorescence microscopy analysis

Leydig cells were incubated with the aromatase inhibitor Letrozole (final concentration 10 ng/ml) or different concentrations of TGF-β1 for 20 h and then fixed with 4% formalin for 30 min at room temperature, rinsed with PBS and permeabilized with 0.1% v/v Triton. Cells were incubated with mouse anti-Cx43 (diluted 1∶200) in PBS containing 1% w/v bovine serum albumin (BSA) overnight at 4°C. After three rinses, cells were incubated at room temperature for 1 h with goat anti-mouse TRITC-conjugated antibodies (1∶100). Finally, cells were mounted in Vecta shield medium with DAPI (Biovalley, Marne-La-Vallée Cedex 3, France) to label nuclei. For negative controls, cover slips were processed without the primary antibody, and no signals were detected. Immunofluorescence images were captured using a Nikon E800 microscope with a Spot-2 camera (Tokyo, Japan).

### Analysis of GJIC

Leydig cells were seeded in a 6-well culture plate overnight. At 70% cell confluence, a GJIC inhibitor Carbenoxolone (Sigma-Aldrich, St. Louis, MO, USA; final concentration 40 µM), aromatase inhibitor Letrozole (Sigma-Aldrich, St. Louis; final concentration 10 ng/ml) or human recombinant TGF-β1 (R&D Systems, Lille, France; final concentration 5 ng/ml) was added. Alternatively, E_2_ (Sigma-Aldrich, St. Louis, MO, USA; final concentration 5 µM) was added 4 h ahead of TGF-β1 exposure. After 20 h of incubation, GJIC was measured by fluorescence recovery after photo-bleaching (FRAP). This method was performed as described previously [37]. Briefly, cells were washed twice with PBS, and then were incubated in culture medium without phenol red, containing 5, 6-carboxyfluorescein diacetate (Research Organics, Ohio, USA) at a final concentration of 50 µg/ml and incubated for 20 min in a 37°C 5% CO_2_ humid incubator. Individual cells were then bleached by strong laser pulses (488 nm 100% and 50 iterations) with a Zeiss confocal microscope LSM 510 (Service Commun de Microscopie, IFR Biomédicale des Saint-Pères, Paris, France). Confocal images were taken every 2 min during a 15 min period after calcein photo-bleaching. Fluorescence recovery was analyzed using LSM software before bleaching, immediately afterwards, and 8 min afterwards. The percentage fluorescence recovery in bleached cells was determined by averaging all cells (n>50) for each experiment.

### Statistical Analysis

All data are expressed as the mean ± SD of three or more independent experiments carried out with different cell preparations. Statistical analysis was performed by using the one-way ANOVA parametric test and significance was accepted at *p*<0.05.

## Results

### Effects of TGF-β1 on E_2_ and T production in Leydig cells

To investigate whether TGF-β1 could influence E_2_ and T production, various concentrations of TGF-β1 (1–10ng/ml) were added to isolated adult Leydig cells for 20 h incubation period (Fig. 1). Compared with the control group, TGF-β1 produced a dose-dependent inhibitory effect on the E_2_ and T secretion of Leydig cells. With increasing concentration TGF-β1 significantly suppressed the basal E_2_ secretion (Fig. 1A) from initial 64 pg/ml to 1 pg/ml with **p<0.01, as well as the basal T secretion (Fig. 1B) from initial 22 ng/ml to 2 ng/ml with **p<0.01.

**Figure 1:** Effects of various concentrations of TGF-β1 on E2 and T production by purified rat Leydig cells. TGF-β1 induced a dose-dependent inhibition of E_2_ as well as T synthesis. Each column represents mean ± S.D of three independent experiments. Significant differences between groups were analyzed with one-way ANOVA. *p<0.05; **p<*0.01* compared with control cells.

### Effects of TGF-β1 on aromatase activity and *Cyp19* expression in Leydig cells

To explore the effect of TGF-β1 on aromatase activity, we next carried out a tritiated water-release assay to address the activity of P450arom. Incubations of Leydig cells were performed in the absence or presence of TGF-β1 for a 20 h period. Although there was no difference between control group and the low dose group (1 ng/ml), when the concentration of TGF-β1 was 2 ng/ml, the activity of aromatase was decreased by 29% in Leydig cells (Fig. 2A). To delineate the mechanism of TGF-β1 inhibition with aromatase activity in Leydig cells, the effect of TGF-β1 on *Cyp19* expressions at the protein and mRNA levels was evaluated. TGF-β1 inhibited *Cyp19* protein expression in a dose-dependent manner (Fig. 2B, C) and the mRNA levels changed in parallel to its protein expression (Fig. 2C). We observed that at 1 ng/ml, TGF-β1 significantly decreased *Cyp19* protein and mRNA levels in Leydig cells from values in the solvent controls and that this inhibitory effect was most significant when the concentration of TGF-β1 was 10 ng/ml.

**Figure 2:** Dose-related effects of TGF-β1 on aromatase activity and Cyp19 expression in purified rat Leydig cells. (A) Inhibition of aromatase activity by pretreatment of Leydig cells with TGF-β1. Cells were serum starved for 24 h and stimulated with TGF-β1 at concentrations between 1 and 10 ng/ml for 20 h. Aromatase activity was evaluated by the tritiated water release assay. The results are expressed as mean ± S.D of three independent experiments (*p<0.05; **p<*0.01*). Significant differences between groups were analyzed with one-way ANOVA. (B) Representative Western blot of *Cyp19* immunoreactivity in Leydig cells, treated for 20 h with TGF-β1 at concentrations between 1 and 10 ng/ml. The β-actin expression is shown as the loading control. (C) The relative amounts of *Cyp19* mRNA (real-time quantitative PCR analysis) and protein (Western blotting analysis) levels in Leydig cells treated with TGF-β1. Data shown are means ± S.D of three independent experiments (*p<*0.05; ## p*<0.01; **p<*0.01*). Significant differences between groups were analyzed with one-way ANOVA.

### Effect of E_2_ and TGF-β1 on Cx43 expression

Cx43 is the major gap junction protein expressed in Leydig cells and has been shown to form functional gap junctions. To determine whether the reduction of E_2_ induced by Letrozole or TGF-β1 could affect Cx43 expression in Leydig cells, the distribution of Cx43 was observed by confocal immunofluorescence microscopy. As shown in Fig. 3A, Cx43 in untreated Leydig cells was predominantly in the form of defined spots uniformly distributed at sites of cell-cell contact and in the cytoplasm. However, a clear decrease in staining intensity of Cx43 in Leydig cells was observed in the presence of the aromatase inhibitor Letrozole. After TGF-β1 exposure for 20 h at the concentration of 1 ng/ml, Cx43 was almost the same as that of control in the pattern of location but distinctly decreased in immunoreactivity in Leydig cells and at the cell borders. The decrease obtained by immunofluorescence staining was confirmed by Western blot analysis. This revealed that the aromatase inhibitor Letrozole and TGF-β1 down-regulated total Cx43 immunoreactivity in Leydig cells (Fig. 3B). This down-regulation was significant when cells were treated with TGF-β1 at concentrations of 2 ng/ml and higher (Fig. 3C).

**Figure 3:** Effects of Letrozole and various concentrations of TGF-β1 on Cx43 expression in purified rat Leydig cells. (A) Subcellular distribution of Cx43 in Leydig cells treated with Letrozole or TGF-β1 observed by confocal microscopy. In untreated cells, Cx43 immunoreactivity is detected both at the cell membrane and in cytoplasm. After treatment with Letrozole or TGF-β1 a distinct decrease of Cx43 immunoreactivity in Leydig cells and at the cell borders is detected. (B) Representative western blot of Cx43 immunoreactivity in Leydig cells, treated for 24 h with Letrozole or TGF-β1 at different concentrations. The β-actin expression is shown as the loading control. (C) The relative amounts of Cx43 protein as shown in (B), demonstrating a significant down-regulation of Cx43 immunoreactivity by TGF-β1 at concentrations of 5 and 10 ng/ml (*p<0.05; **p<*0.01*). Significant differences between groups were analyzed with one-way ANOVA.

### Effect of E_2_ and TGF-β1 on GJIC between Leydig cells

Since Cx43 is the major functional protein forming gap junction channels in Leydig cells and plays critical role in regulating gap junction communication, we investigated if GJIC of Leydig cells is affected by E_2_ and TGF-β1. The results showed that Carbenoxolone, an established GJIC inhibitor, reduced the dye transfer rate by almost 90% (Fig. 4A, B). This result serves as a positive control for the reliability of the gap-FRAP technique to measure changes in GJIC [38]. Compared with PBS-treated cells, the transfer rate of the fluorescent dye 5, 6-carboxylfluorescein diacetate was significantly lower in both Letrozole- and TGF-β1-treated Leydig cells (Fig. 4A, B). However, the TGF-β1-induced down-regulation of GJIC was attenuated when the cells were treated with E_2_ before the addition of TGF-β1 (Fig. 4).

**Figure 4:** FRAP analysis of GJIC in Leydig cells. (A) Effects of various treatments on dye transfer in Leydig cells. Left panel: Image of the target cell before bleaching (white collar). Middle panel: Image of the target cell after bleaching. Right panel: Image of the target cell after 8 min of fluorescence recovery. Recovery of fluorescence in the target cell was caused by influx of dye from adjacent cells. NC: In normal control group, cells were treated with phosphate-buffered saline; Carbenoxolone: cells were treated with 40 µM Carbenoxolone for 20 h; Letrozole: cells were treated with Letrozole of 10 ng/ml for 20 h; TGF-β1: cells were treated with 5 ng/ml TGF-β1 for 20 h; E_2_: cells were treated with 5 µM E_2_ for 4 h and 5 g/ml TGF-β1 for 20 h. (B) Histograms representing the percentage of GJIC in each condition (*p<0.05; **p<*0.01*). Significant differences between groups were analyzed with one-way ANOVA.

## Discussion

The results from the present study showed that TGF-β1 down-regulated the level of E_2_ secretion, the activity of P450arom and the expression of *Cyp19* in adult rat Leydig cells. Such reduction of E_2_ could explain the dysfunction of Cx43-mediated GJIC between Leydig cells treated with TGF-β1, since E_2_ restored the TGF-β1 inhibition of GJIC. These unique effects of TGF-β1 imply that it may have novel functions in the testis, moderating the intercellular communication between Leydig cells.

The main source of estrogen in the testis is conversion of androgen catalyzed by P450arom. Leydig cells have been demonstrated to be a major site of aromatase expression in the adult testis [8]. In this study we demonstrated that TGF-β1 treatment decreased E_2_ and T production, as well as aromatase activity in Leydig cells, in a dose-dependent manner, and in parallel decreased expression of *Cyp19* mRNA and protein was also observed. Interestingly, TGF-β1 reduced E_2_ synthesis significantly at the concentration of 1 ng/ml but had no effect on P450arom activity at the same concentration. This observation suggests that the production of E_2_ may well be the sum of decreased T and reduced aromatase expression. These findings concur with those obtained in germ cells, where TGF-β1 significantly inhibits aromatase activity and P450arom transcripts [39]. In addition, it has been demonstrated that TGF-β1 inhibits E_2_ production in cultured human trophoblast cells [40], human fetal hepatocytes [41], and skin fibroblasts [42]. Although the mechanism by which TGF-β1 exerts its inhibitory effect on aromatase gene expression in Leydig cells remains to be established, one possible explanation is transcriptional regulation of *Cyp19*. Expression of P450arom in rat testicular cells is controlled primarily by promoter PII, proximal to the translation start site [43]. It has been proved that TGF-β1 inhibits the promoter activity via the Smad2 signalling pathway in human trophoblast cells [44]. Moreover, the orphan receptor steroidogenic factor-1 (SF-1) binding site has been identified as the response element in the proximal promoter PII of the rat aromatase gene [45], and TGF-β1 has been proved to inhibit SF-1 expression both at the transcriptional and translational levels in the mouse adrenocortical cell Y-1 [46] and human adrenocortical cell H295R [47].

It has been proved that stimulation of testosterone production by hCG is associated with a decrease in Cx43 mRNA levels in Leydig cells both in vitro and in vivo [48]. Given that Leydig cells are the main site of conversion of androgens into estrogens in the testis, and that GJ-protein expression is regulated in part by steroid hormones in steroid-sensitive organs, it is essential to investigate whether there is a correlation between E_2_ synthesized by Leydig cells and Cx43-mediated intercellular communication. In the present study, we showed that administration of Letrozole or TGF-β1 to rat Leydig cells decreased Cx43 expression and down regulated GJIC. Considering that both Letrozole and TGF-β1 inhibit E_2_ production by Leydig cells, it is possible that E_2_ operates as a local regulator in the fine-tuning of the gap junction between Leydig cells. Recent studies demonstrate that the expression of Cx43 is greatly reduced by ovariectomy and is restored by treatment with estrogen [49]. Also, GJ coupling and the amount of Cx43 protein are reduced after anti-estrogen treatment in bovine myocytes from the circular layer of myometrium [50]. One possible explanation for these results is the regulation of transcripts encoding Cx43 by estrogen. Activated ERs are transcription factors that bind to estrogen response elements (EREs) in the regulatory region of target genes. Two related estrogen receptors ERα and ERβ have been demonstrated to be expressed in rat Leydig cells [51]; and a series of half- palindromic EREs is present in the promoter of the rat connexin43 gene [45], [52], [53]. Transcription of Cx43 can be induced by estrogen via an ER-dependent pathway during preimplantation [54]. Therefore, estrogen may increase Cx43 through a genomic pathway mediated by the nuclear receptors in rat Leydig cells. Although TGF-β1 distinctively down-regulated gap junctional communication between Leydig cells, prior addition of estradiol to the culture medium attenuated this inhibition to an extent. Up-regulation of cell-to-cell communication and Cx43 expression by estrogen has been observed in the human myometrium [26], similarly, in rat cardiomyocytes, estrogen has been shown to increase GJIC via ER-mediated signalling at a pharmacological concentration [55]–[56]. Since Cx43 is a gap junctional protein expressed in Leydig cells, we speculate that E_2_ modulates GJIC in Leydig cells through ER/Cx43 pathway.

In conclusion, the present study demonstrates that TGF-β1 has a significant inhibitory effect on estrogen production by rat Leydig cells possibly via down-regulation of aromatase gene expression and activity. This could decrease Cx43 expression, leading to Cx43-mediated gap junction between Leydig cells. Future studies are required to clarify further the mechanisms of regulation of E_2_ in the gap junctions between Leydig cells.
